The article "Methylation-induced downregulation and tumor suppressive role of microRNA-29b in gastric cancer through targeting LASP1" was retracted in 2023. Reasons: duplicated images; signs of a paper mill; concerns about the data.

# Methylation-induced downregulation and tumor suppressive role of microRNA-29b in gastric cancer through targeting LASP1

**DOI:** 10.18632/oncotarget.21431

**Published:** 2017-09-30

**Authors:** Hui Li, Guoqing Liu, Ke Pan, Xiongying Miao, Yong Xie

**Affiliations:** ^1^ Department of Anesthesia, Second Xiangya Hospital, Central South University, Changsha, Hunan, China; ^2^ Department of General Surgery, Second Xiangya Hospital, Central South University, Changsha, Hunan, China

**Keywords:** gastric cancer, microRNA, methylation, LIM and SH3 protein 1

## Abstract

MicroRNAs (miRs) have been demonstrated to play promoting or tumor suppressive roles in various human cancers, but the regulatory mechanism of miR-29b underlying gastric cancer development and progression still remains largely unclear. In the present study, we found that miR-29b was significantly downregulated in gastric cancer tissues and cell lines. Low expression of miR-29b was significantly associated with DNA methylation, and treatment with DNA methyltransferase inhibitor 5-Aza-20-deoxycytidine upregulated miR-29b in gastric cancer cells. In addition, both reduced miR-29b expression and miR-29b methylation were associated with disease progression and poor prognosis in gastric cancer. Restoration of miR-29b caused a reduction in gastric cancer cell proliferation, migration, and invasion, and inhibited tumor growth *in vivo*. LASP1 was then identified as a target gene of miR-29b in gastric cancer cells. Moreover, upregulation of LASP1 was significantly associated with gastric cancer progression and poor prognosis. Knockdown of LASP1 also suppressed the proliferation, migration, and invasion of gastric cancer cells. Moreover, overexpression of LASP1 impaired the suppressive effects of miR-29b on the malignant phenotypes of gastric cancer cells, suggesting that miR-29b may inhibit gastric cancer growth and metastasis via targeting LASP1. According to these data, miR-29b may be used as a potential therapeutic candidate for gastric cancer.

## INTRODUCTION

Gastric cancer is one of the most common human malignant tumors, associated with high morbidity and mortality worldwide [1]. As the development of gastric cancer is a multistep and multifactorial process, investigation on the underlying mechanism during gastric cancer growth and metastasis seems to be benefit for the development of effective therapeutic strategies for gastric cancer [2–4].

MicroRNAs (miRs) are a kind of 18-25 nucleotides in length non-coding RNAs, and act as key regulators for gene expression [5]. They could directly bind to the 3’-untranslational region (UTR) of their target mRNAs, and cause translation inhibition or mRNA degradation [6, 7]. Through inhibiting the expression of their targets, miRs participate in the regulation of various cellular biological processes, such as cell growth, proliferation, differentiation, apoptosis, cell cycle progression, and tumorigenesis [5, 6, 8]. Recent studies have shown that many miRs play suppressive or oncogenic roles in gastric cancer including miR-126 [9], miR-145 [10], miR-326 [4], miR-506 [11], and miR-29 [12].

The article "Methylation-induced downregulation and tumor suppressive role of microRNA-29b in gastric cancer through targeting LASP1" was retracted in 2023. Reasons: duplicated images; signs of a paper mill; concerns about the data.

MiR-29b has previously been implicated in some physiological and pathological processes [13, 14]. For instance, miR-29b could inhibit the migration and proliferation of vascular smooth muscle cells in neointimal formation[15]. Besides, miR-29b is involved in the development of Alzheimer disease through regulating the expression of BACE1 [16]. In recent years, the tumor suppressive effect of miR-29b has been gradually reported in some common human cancers including gastric cancer [14, 17, 18]. For instance, Zhang et al. reported that miR-29b could target AKT2 to inhibit the invasion of gastric cancer cells [18]. Kong et al. showed that miR-29b had suppressive effects on the proliferation and migration of gastric cancer cells by inhibition of KDM2A [19]. Besides, miR-29b could reduce the cisplatin resistance of gastric cancer cells by directly targeting PI3K/Akt pathway [20]. However, whether other targets of miR-29b exist in gastric cancer still needs to be studied.

Accordingly, we mainly aimed to explore the regulatory mechanism of miR-29b underlying gastric cancer development and progression.

## RESULTS

### MiR-29b is downregulated in gastric cancer

To reveal the function of miR-29b in gastric cancer, real-time PCR was conducted to examine the miR-29b expression in gastric cancer tissues and adjacent non-tumor tissues. As shown in Figure 1A, miR-29b was significantly downregulated in gastric cancer tissues compared with adjacent non-tumor tissues.

**Figure 1:** High methylation contributes to the downregulated of miR-29b in gastric cancer **(A)** Real-time RT-PCR was conducted to examine the miR-29b expression levels in 84 cases gastric cancer tissues and adjacent non-tumor tissues. **(B)** The gastric cancer patients with low expression of miR-29b showed shorter survival time when compared with those with high miR-29b expression. **(C)** Real-time RT-PCR was conducted to examine the miR-29b expression levels in human gastric cancer cell lines (AGS, BGC-823, SGC-7901, and MGC-803) compared with normal human gastric mucosa epithelial cell line GES-1. ^**^ P<0.01 vs. GES-1. **(D)** Methylation-specific PCR was conducted to examine the methylation status of miR-29b in human gastric cancer cell lines (AGS, BGC-823, SGC-7901, and MGC-803) and normal human gastric mucosa epithelial cell line GES-1. **(E)** Gastric cancer cell lines were treated with DNA methyltransferase inhibitor 5-aza for 48 h, and real-time RT-PCR was conducted to examine the expression levels of miR-29b. Untreated gastric cancer cell lines were used as control group. ^**^ P<0.01 vs. untreated. Data were expressed as the group means ± SD.

The article "Methylation-induced downregulation and tumor suppressive role of microRNA-29b in gastric cancer through targeting LASP1" was retracted in 2023. Reasons: duplicated images; signs of a paper mill; concerns about the data.

The clinical significance of miR-29b expression in gastric cancer was further studied. Our data indicated that low miR-29b expression was significantly associated with poor differentiation, lymph node metastasis, and advanced clinical stage in gastric cancer, suggesting that the miR-29b downregulation may contribute to gastric cancer progression (Table 1). Moreover, the gastric cancer patients with low expression of miR-29b showed shorter survival time, when compared with those with high miR-29b expression, suggesting that the downregulation of miR-29b is associated with poor prognosis (Figure 1B).

**Table 1:** Association between miR-29b expression and clinicopathologic characteristics of gastric cancer patients

Variables	Cases (n=84)	Low expression (n=44)	High expression (n=40)	P value
**Age (years old)**				0.828
≤65	37	20	17	
≤65	47	24	23	
**Sex**				0.656
Male	51	28	23	
Female	33	16	17	
**Tumor differentiation**				0.017^*^
Well and Moderate	45	18	27	
Poor	39	26	13	
**Tumor size (cm)**				0.165
≤5	56	26	30	
≤5	28	18	10	
**Lymph node metastasis**				0.018^*^
Present	41	27	14	
Absent	43	17	26	
**Distant metastasis**				0.055
Present	16	12	4	
Absent	68	32	36	
**TNM stage**				0.005^**^
I-II	43	16	27	
III-IV	41	28	13	

^*^P<0.05; ^**^ P<0.01.

In addition, the expression of miR-29b in gastric cancer cell lines was examined. As indicated in Figure 1C, miR-29b was also significantly downregulated in gastric cancer cell lines including AGS, BGC-823, SGC-7901, and MGC-803, when compared with that in normal human gastric mucosa epithelial GES-1 cells. Taken together, miR-29b is downregulated in gastric cancer.

### High methylation contributes to the downregulated of miR-29b in gastric cancer

We further investigated the molecular mechanism underlying miR-29b expression in gastric cancer tissues and cell lines. The methylation status of miR-29b in gastric cancer tissues and adjacent non-tumor tissues was examined in using methylation-specific PCR (MSP). We observed that 52 gastric cancer tissues showed methylated miR-29b, while only 6 adjacent non-tumor tissues showed methylated miR-29b (P<0.0001). Moreover, high methylation of miR-29b was also associated with the malignant progression of gastric cancer (Table 2).

**Table 2:** Association between miR-29b methylation status and clinicopathologic characteristics of gastric cancer patients

Variables	Cases (n=84)	Methylated (n=52)	Unmethylated (n=32)	P value
**Age (years old)**				0.498
≤65	37	21	16	
≤65	47	31	16	
**Sex**				0.646
Male	51	33	18	
Female	33	19	14	
**Tumor differentiation**				0.042^*^
Well and Moderate	45	23	22	
Poor	39	29	10	
**Tumor size (cm)**				0.099
≤5	56	31	25	
≤5	28	21	7	
**Lymph node metastasis**				0.014^*^
Present	41	31	10	
Absent	43	21	22	
**Distant metastasis**				0.092
Present	16	13	3	
Absent	68	39	29	
**TNM stage**				0.004^**^
I-II	43	20	23	
III-IV	41	32	9	

^*^ P<0.05; ^**^ P<0.01.

The article "Methylation-induced downregulation and tumor suppressive role of microRNA-29b in gastric cancer through targeting LASP1" was retracted in 2023. Reasons: duplicated images; signs of a paper mill; concerns about the data.

Similarly, the gastric cancer cell lines (AGS, BGC-823, SGC-7901, and MGC-803) showed positive methylation status, but no methylation was detected in normal human gastric mucosa epithelial GES-1 cells (Figure 1D). To further confirm that high methylation contributes to miR-29b inhibition in gastric cancer cells, these gastric cancer cell lines were treated with DNA methyltransferase inhibitor 5-aza for 48 h. After treatment, we observed a significant increase in the miR-29b expression in these gastric cancer cell lines (Figure 1E). These data indicates that the downregulation of miR-29b is partly at least due to the high methylation in gastric cancer cells.

### Overexpression of miR-29b inhibits gastric cancer cell growth *in vitro* and *in vivo*

We further investigated the regulatory effects of miR-29b on the growth of gastric cancer cells *in vitro* and *in vivo*. AGS and BGC-823 cells were transfected with miR-29b mimic or miR-NC mimic, respectively. After transfection, the miR-29b levels were significantly increased in the miR-29b group compared with miR-NC group (Figure 2A). MTT assay data further indicated that the proliferation of gastric cancer cells was significantly reduced in the miR-29b group compared with miR-NC group, suggesting that miR-29b has suppressive effects on gastric cancer cell proliferation (Figure 2B). After that, the pYr-LVX-miR-29b or pYr-LVX-miR-NC lentiviral plasmid was then stably transfected into AGS and BGC-823 cells, which were then subcutaneously implanted into the nude mice. All mice were sacrificed on 60 days after implantation, and the tumor xenograft were obtained (Figure 2C). The tumor weight and volume were significantly reduced in the miR-29a group when compared to the miR-NC group (Figure 2D-2E). Taken together, miR-29b overexpression inhibits gastric cancer cell growth *in vitro* and *in vivo*.

**Figure 2:** Overexpression of miR-29b inhibits gastric cancer cell growth *in vitro* and *in vivo* AGS and BGC-823 cells were transfected with miR-29b mimic or miR-NC mimic, respectively. **(A)** Real-time RT-PCR was conducted to examine the miR-29b expression levels. **(B)** MTT was conducted to examine cell proliferation. After that, the pYr-LVX-miR-29b or pYr-LVX-miR-NC lentiviral plasmid was then stably transfected into AGS and BGC-823 cells, which were then subcutaneously implanted into the nude mice. **(C)** All mice were sacrificed on 60 days after implantation, and the tumor xenograft were obtained. **(D)** Tumor weight and **(E)** volume were examined. ^**^ P<0.01 vs. miR-NC. Data were expressed as the group means ± SD.

The article "Methylation-induced downregulation and tumor suppressive role of microRNA-29b in gastric cancer through targeting LASP1" was retracted in 2023. Reasons: duplicated images; signs of a paper mill; concerns about the data.

### MiR-29b has suppressive effects on the migration and invasion of gastric cancer cells

We then studied the potential effects of miR-29b on gastric cancer cell migration and invasion by using wound healing assay and transwell assay. Our data indicated that the migration and invasion of AGS and BGC-823 cells were significantly reduced in the miR-29b group compared with the miR-NC group, indicating that MiR-29b has suppressive effects on the migration and invasion of gastric cancer cells (Figure 3).

**Figure 3:** Overexpression of miR-29b inhibits gastric cancer cell migration and invasion AGS and BGC-823 cells were transfected with miR-29b mimic or miR-NC mimic, respectively. **(A)** Wound healing assay was conducted to examine the cell migration. **(B)** Transwell assay was conducted to examine the cell invasion. ^**^ P<0.01 vs. miR-NC. Data were expressed as the group means ± SD. Magnification for wound healing assay:40x. Magnification for transwell assay: 400x.

### LASP1 is a target gene of miR-29b in gastric cancer cells

Bioinformatics analysis data showed that LASP1 was a potential target of miR-29b. To clarify their relationship, we firstly studied the effect of miR-29b upregulation or downregulation on the expression of LASP1 in gastric cancer cells. As shown in Figure 4A-4B, the mRNA and protein expression of LASP1 were significantly downregulated in gastric cancer cells after overexpression of miR-29b. To further confirm these findings, AGS and BGC-823 cells were transfected with miR-29b inhibitor or NC inhibitor respectively. After transfection, the miR-29b levels were significantly reduced in the miR-29b inhibitor group compared with NC inhibitor group (Figure 4C). We then showed that transfection with miR-29b inhibitor significantly increased the mRNA and protein expression of LASP1 in AGS and BGC-823 cells, when compared with the NC inhibitor group (Figure 4D-4E). Therefore, LASP1 is negatively regulated by miR-29b in gastric cancer cells.

**Figure 4:** The expression of LASP1 was negatively mediated by miR-29b in gastric cancer cells AGS and BGC-823 cells were transfected with miR-29b mimic or miR-NC mimic, respectively. After transfection, **(A)** real-time PCR and **(B)** western blot were performed to determine the mRNA and protein expression of LASP1. For (A-B)^**^ P<0.01 vs. miR-NC. After that, AGS and BGC-823 cells were transfected with miR-29b inhibitor or NC inhibitor, respectively. **(C)** After transfection, real-time PCR was conducted to examine the miR-29b expression. Then, **(D)** real-time PCR and **(E)** western blot were used to examine the mRNA and protein levels of LASP1. For (C-E) ^**^ P<0.01 vs. NC inhibitor. Data were expressed as the group means ± SD.

The article "Methylation-induced downregulation and tumor suppressive role of microRNA-29b in gastric cancer through targeting LASP1" was retracted in 2023. Reasons: duplicated images; signs of a paper mill; concerns about the data.

To further confirm whether LASP1 is a direct target gene of miR-29b in gastric cancer, the pGL3-LASP1-3’UTR and pGL3-LASP1-mut 3’UTR luciferase reporter plasmids were generated (Figrue 5A-5B). We then performed dual luciferase reporter gene assay in AGS and BGC-823 cells. Our data showed that the luciferase activity was decreased in cells co-transfected with miR-29b mimics and pGL3-LASP1-3’UTR luciferase reporter plasmid, which was eliminated by transfection with the pGL3-LASP1-mut 3’UTR luciferase reporter plasmid (Figure 5C-5D). Therefore, miR-29b can directly bind to the 3’UTR of LASP1 mRNA in gastric cancer cells.

**Figure 5:** LASP1 is a target gene of miR-29b in gastric cancer cells **(A)** Targetscan data indicate that LASP1 is a putative target gene of miR-29b. **(B)** pGL3-LASP1-3’UTR and pGL3-LASP1-mut 3’UTR luciferase reporter plasmids were generated. **(C)** Luciferase reporter gene assay was conducted using AGS and BGC-823 cells. ^**^ P<0.01 vs. Control. Data were expressed as the group means ± SD.

### LASP1 is significantly upregulated in gastric cancer

We further examined the expression of LASP1 in gastric cancer tissues and cell lines. Our data showed that the mRNA and protein levels of LASP1 were significantly higher in gastric cancer tissues compared with adjacent non-tumor tissues (Figure 6A and 6B). Interestingly, we observed an inverse correlation between the miR-29b and LASP1 expression in gastric cancer tissues (Figure 6C), suggesting that the upregulation of LASP1 may be due to the downregulation of miR-29b in gastric cancer.

**Figure 6:** LASP1 is significantly upregulated in gastric cancer **(A)** Real-time RT-PCR and **(B)** western blot were conducted to examine the mRNA and protein expression of LASP1 in 84 cases gastric cancer tissues and adjacent non-tumor tissues. **(C)** An inverse correlation between the miR-29b and LASP1 expression in gastric cancer tissues. **(D)** The gastric cancer patients with high expression of LASP1 showed shorter survival time when compared with those with low LASP1 expression. **(E)** Real-time PCR and **(F)** western blot were performed to determine the mRNA and protein expression of LASP1 in human gastric cancer cell lines (AGS, BGC-823, SGC-7901, and MGC-803) compared with normal human gastric mucosa epithelial cell line GES-1. For (E-F) ^**^ P<0.01 vs. GES-1. Data were expressed as the group means ± SD.

The article "Methylation-induced downregulation and tumor suppressive role of microRNA-29b in gastric cancer through targeting LASP1" was retracted in 2023. Reasons: duplicated images; signs of a paper mill; concerns about the data.

Moreover, the expression of LASP1 was significantly associated with the tumor size, metastasis, TNM stage in gastric cancer (Table 3), as well as shorter survival time of patients (Figure 6D). Moreover, according to the result of multivariate analysis, low miR-29b expression and high LASP1 expression was not independent association with worse prognosis of GCs (Table 4). However, it still supports miR-29b and LASP1 expression as risk factors (HR>1) for patient survival (Table 4). In addition, the mRNA and protein levels of LASP1 were also increased in gastric cancer cell lines compared with GES-1 cells (Figure 6E-6F). Based on the above findings, we suggest that the upregulation of LASP1 may be due to the downregulation of miR-29b, which further contributes to the malignant progression and poor prognosis in gastric cancer.

**Table 3:** Association between LASP1 expression and clinicopathologic characteristics of gastric cancer patients

Variables	Cases (n=84)	Low expression (n=45)	High expression (n=39)	P value
**Age (years old)**				0.663
≤65	37	21	16	
≤65	47	24	23	
**Sex**				0.372
Male	51	25	26	
Female	33	20	13	
**Tumor differentiation**				0.125
Well and Moderate	45	28	17	
Poor	39	17	22	
**Tumor size (cm)**				0.036^*^
≤5	56	35	21	
≤5	28	10	18	
**Lymph node metastasis**				0.016^*^
Present	41	16	25	
Absent	43	29	14	
**Distant metastasis**				0.013^*^
Present	16	4	12	
Absent	68	41	27	
**TNM stage**				0.004^**^
I-II	43	30	13	
III-IV	41	15	26	

^*^ P<0.05; ^**^ P<0.01.

**Table 4:** Multivariate analysis for overall survival of gastric cancer patients

Variables	HR	CI (95%)	P value
Tumor differentiation	1.172	0.766-1.747	0.471
Tumor size	1.431	0.896-2.282	0.132
Lymph node metastasis	1.813	0.867-3.724	0.102
Distant metastasis	1.878	0.934-3.771	0.072
TNM stage	2.048	1.302-3.215	0.004^**^
miR-29b expression	1.514	0.977-2.646	0.114
LASP1 expression	1.488	0.922-2.397	0.12

^**^ P<0.01.

### Knockdown of LASP1 inhibits the malignant phenotypes of gastric cancer cells

As LASP1 was significantly upregulated in gastric cancer, AGS and BGC-823 cells were transfected with LASP1 siRNA to knockdown its expression. After transfection, the mRNA and protein levels of LASP1 were significantly decreased in the LASP1 siRNA group compared with the NC siRNA group (Figure 7A-7B). Further investigation showed that the proliferation, migration and invasion of cells were significantly downregulated in the LASP1 siRNA group compared with the NC siRNA group, suggesting that LASP1 plays a promoting role in regulating the proliferation, migration and invasion of gastric cancer cells (Figure 7C-7E).

The article "Methylation-induced downregulation and tumor suppressive role of microRNA-29b in gastric cancer through targeting LASP1" was retracted in 2023. Reasons: duplicated images; signs of a paper mill; concerns about the data.

**Figure 7:** Knockdown of LASP1 inhibits the malignant phenotypes of gastric cancer cells AGS and BGC-823 cells were transfected with LASP1 siRNA or NC siRNA, respectively. After transfection, **(A)** real-time PCR and **(B)** western blot were performed to determine the mRNA and protein expression of LASP1. Then, **(C)** MTT assay, **(D)** wound healing assay and **(E)** transwell assay were conducted to examine the cell proliferation, migration and invasion, respectively. ^**^ P<0.01 vs. NC siRNA. Data were expressed as the group means ± SD. Magnification for wound healing assay:40x. Magnification for transwell assay: 400x.

### Overexpression of LASP1 impaired the suppressive effects of miR-29b on the proliferation, migration, and invasion of gastric cancer cells

After that, we further investigated whether LASP1 was involved in the miR-29b-malignant phenotypes of gastric cancer cells. MiR-29b-overexpressing AGS and BGC-823 cells were transfected with pcDNA3.1-LASP1 ORF plasmid or blank pcDNA3.1 vector, respectively. After transfection, the mRNA and protein levels of LASP1 were significantly increased in the miR-29b+LASP1 group compared with miR-29b+blank group (Figrue 8A-8B). MTT assay, wound healing assay and transwell assay data further showed that the cell proliferation, migration, and invasion were also increased in the miR-29b+LASP1 group compared with the miR-29b+blank group (Figure 8C-8E). These findings demonstrate that LASP1 overexpression impaired the suppressive effects of miR-29b on the proliferation, migration, and invasion of gastric cancer cells.

**Figure 8:** Overexpression of LASP1 impaired the suppressive effects of miR-29b on the proliferation, migration, and invasion of gastric cancer cells MiR-29b-overexpressing AGS and BGC-823 cells were transfected with pcDNA3.1-LASP1 plasmid or blank pcDNA3.1 vector, respectively. After transfection, (A) real-time PCR and (B) western blot were performed to determine the mRNA and protein expression of LASP1. Then, (C) MTT assay, (D) wound healing assay and (E) transwell assay were conducted to examine the cell proliferation, migration and invasion, respectively. ^**^ P<0.01 vs. miR-29b+blank. Data were expressed as the group means ± SD. Magnification for wound healing assay:40x. Magnification for transwell assay: 400x.

## DISCUSSION

The molecular mechanism of miR-29b underlying gastric cancer development and progression remains largely unclear. Here we found that miR-29b was significantly downregulated in gastric cancer. Low expression of miR-29b was significantly associated with DNA methylation, and treatment with DNA methyltransferase inhibitor upregulated its expression in gastric cancer cells. Besides, both miR-29b methylation and low miR-29b expression were associated with disease progression and poor prognosis in gastric cancer. Restoration of miR-29b caused a reduction in gastric cancer cell proliferation, migration, and invasion, and inhibited tumor growth *in vivo*. LASP1 was then identified as a target gene of miR-29b in gastric cancer cells. Moreover, upregulation of LASP1 was significantly associated with gastric cancer progression and poor prognosis. Knockdown of LASP1 also suppressed the proliferation, migration, and invasion of gastric cancer cells. In addition, overexpression of LASP1 impaired the suppressive effects of miR-29b on the malignant phenotypes of gastric cancer cells.

The article "Methylation-induced downregulation and tumor suppressive role of microRNA-29b in gastric cancer through targeting LASP1" was retracted in 2023. Reasons: duplicated images; signs of a paper mill; concerns about the data.

In recent years, the different roles of miRs in gastric cancer have been widely studied. For instance, miR-187 promotes growth and metastasis of gastric cancer by inhibiting FOXA2 [21]. MiR-218 inhibits proliferation, migration, and EMT of gastric cancer cells by targeting WASF3 [3]. Recently, genetic variation in miR-29 has been suggested to have a critical role in genetic susceptibility to gastric cancer, and miR-29b has been demonstrated to play a suppressive role in gastric cancer [22]. Several target genes of miR-29b have been identified in gastric cancer, such as KDM2A [19] and AKT2 [18]. In this study, we found that miR-29b was significantly downregulated in gastric cancer tissues and cell lines, consistent with previous findings [23].

Moreover, we found that the methylation status of miR-29b was significantly higher in gastric cancer tissues and cell lines. We speculated that the high methylation status may be a main cause for the downregulation of miR-29b in gastric cancer. To verify this speculation, we used DNA methyltransferase inhibitor to treat gastric cancer cells. After treatment, the miR-29b levels were significantly increased, which confirmed our speculation. In fact, it has been reported a crucial crosstalk between miR-29b and DNMT3A/3B via a double-negative feedback loop. MiR-29b could directly target DNMT3A/3B, and thus inhibit their expression, while DNMT3A/3B could also inhibit the expression of miR-29b via CpG island promoter hypomethylation [24]. Besides, Cui et al. reported that deregulation between miR-29b and DNMT3A was associated with the downregulation of CDH1, which further promoted gastric cancer cell migration and invasion [25]. Therefore, the downregulation of miR-29b in gastric cancer may be associated with DNMT3A/3B.

The article "Methylation-induced downregulation and tumor suppressive role of microRNA-29b in gastric cancer through targeting LASP1" was retracted in 2023. Reasons: duplicated images; signs of a paper mill; concerns about the data.

As the clinical significance of miR-29b expression in gastric cancer has never previously been reported, we further study it and showed that both low miR-29b expression and miR-29b methylation were significantly associated with the poor differentiation and lymph node metastasis in gastric cancer, suggesting that the downregulation of miR-29b may contribute to gastric cancer progression. As we then found that overexpression of miR-29b inhibited the proliferation, migration and invasion of gastric cancer cells *in vitro* and tumor growth *in vivo*, we suggest that miR-29b may be used as a potential therapeutic candidate for gastric cancer.

After that, we investigated the potential target genes of miR-29b in gastric cancer. Through bioinformatics prediction, we found that LASP1 was a potential target gene of miR-29b, and the targeting relationship between miR-29b and LASP1 was evolutionally conserved. LASP1, a member of LIM proteins and of the nebulin family of actin-binding proteins, is a cAMP and cGMP dependent signaling protein, and can bind to the actin cytoskeleton at extensions of the cell membrane [26]. Recent studies have revealed that LASP1 was frequently upregulated in malignant tumors and functioned as an oncogene in gastric cancer [27]. Zheng et al. reported that LASP-1 was upregulated in gastric cancer tissues, and its expression was significantly associated with tumor size, invasive depth, TNM stage, lymph node metastasis, as well as poor prognosis of gastric cancer patients [27], consistent with our data. Moreover, Wang et al. demonstrated that miR-218 inhibited the proliferation, migration, and invasion and promotes apoptosis of gastric cancer cells by targeting LASP1 [28]. However, whether other miRs directly target LASP1 in gastric cancer has not previously been reported. In this study, we identified LASP1 as a novel target of miR-29b by using luciferease reporter gene assay, and the expression of LASP1 was negatively regulated by miR-29b in gastric cancer cell lines. After that, we investigated the molecular mechanism of LASP1 in regulating the malignant phenotypes of gastric cancer cells, and our data indicated that inhibition of LASP1 effectively reduced the proliferation, migration and invasion of gastric cancer cells, consistent with previous data [27]. Since we had found that LASP1 was a target gene of miR-29b in gastric cancer cells, we speculated that LASP1 might be involved in the miR-29b-mediated malignant phenotypes of gastric cancer cells, and our data confirmed this speculation that overexpression of LASP1 impaired the inhibitory effects of miR-29b on gastric cancer cells.

In summary, this is the first study demonstrating that miR-29b is downregulated in gastric cancer due to DNA methylation, and acts as a tumor suppressor partly at least via directly targeting LASP1. Our findings expand the understanding of the regulatory mechanism of miRs in human cancers.

The article "Methylation-induced downregulation and tumor suppressive role of microRNA-29b in gastric cancer through targeting LASP1" was retracted in 2023. Reasons: duplicated images; signs of a paper mill; concerns about the data.

## MATERIALS AND METHODS

### Tissue collection

This study was approved by the Ethic Committee of Second Xiangya Hospital, Central South University, Changsha, China. A total of 84 primary gastric cancer tissues and adjacent non-tumor tissues were collected from our hospital between October, 2009 to April, 2011. These gastric cancer patients included 51 male and 33 female from 37 to 83 years old, with mean of 66.5 years old. All informed consents were obtained. The clinical information of these patients was summarized in Table 1. No patients received radiation therapy or chemotherapy before surgical resection. After surgical resection, the tissues were immediately snap-frozen and stored in liquid nitrogen before use.

### Cell culture

Human gastric cancer cell lines including AGS, BGC-823, SGC-7901, and MGC-803, and normal human gastric mucosa epithelial cell line GES-1 were purchased from ATCC, USA. Cells were cultured in DMEM (Thermo Fisher, USA) supplemented with 10% fetal bovine serum (FBS, Thermo Fisher) in a 37°C humidified atmosphere of 5% CO2.

### Reverse transcription-quantitative polymerase chain reaction (RT-qPCR)

Total RNA was extracted using Trizol Reagent (Thermo Fisher), and then converted into cDNA using using Reverse Transcription Kit (Thermo Fisher). Reverse transcription was performed at 16°C for 30 min, followed by an incubation at 42°C for 30 min and enzyme inactivation at 85°C for 5 min. For miR expression, real-time PCR was performed using miRNA Q-PCR Detection Kit (GeneCopoeia, Rockville, MD, USA) on ABI 7500 thermocycler (Thermo Fisher). For mRNA expression detection, real-time PCR was performed using SYBR Green I Real-Time PCR kit (Biomics, Nantong, China) on ABI 7500 thermocycler. U6 and GAPDH were used as internal references, respectively. The primers used for miR-29b and its reference gene U6 were purchased from Fulengen (Guangzhou, China), and the sequences were not supplied by the manufacturer. The specific primer pairs for LASP1 were forward, 5’- TGCGGCAAGATCGTGTATCC -3’ and reverse, 5'- GCAGTAGGGCTTCTTCTCGTAG -3’. The specific primer pairs for GAPDH were forward 5’- GGAGCGAGATCCCTCCAAAAT -3’ and reverse 5’- GGCTGTTGTCATACTTCTCATGG -3’. The PCR reaction condition was 95°C for 3 min, followed by 40 cycles of denaturation at 95°C for 15 sec and annealing/elongation step at 60°C for 30 sec. The relative expression was analyzed by the 2^-ΔΔCt^ method [29].

### Measurement of miR-29b promoter CpG island methylation status by MSP

Genomic DNA was extracted using the TIANamp Genomic DNA Kit (Tiangen, Beijing, China) , according to the manufacturer's instruction, and 1 μg of genomic DNA was modified with bisulfite using the EZ DNA Methylation-Gold™ Kit (ZYMO RESEARCH, CA, USA), according to the manufacturer's instruction. MSP was performed on bisulfate-treated DNA. The primers used for methylated miR-29b was 5’-TCGCAGAGGATTAGACAGAG-3’ and 5’-AGGGATTTCACAACGTTCAT-3’. The PCR reaction condition was 95°C for 3 min, followed by 30 cycles of denaturation at 95°C for 15 sec, annealing at 60°C for 30 sec and elongation step at 72°C for 30 sec. PCR amplification data were analyzed by using gel electrophoresis.

The article "Methylation-induced downregulation and tumor suppressive role of microRNA-29b in gastric cancer through targeting LASP1" was retracted in 2023. Reasons: duplicated images; signs of a paper mill; concerns about the data.

### Cell transfection

AGS and BGC-823 cells were transfected with scramble miR (miR-NC), miR-29b mimics, negative control (NC) inhibitor, miR-29b inhibitor, LASP1 siRNA, NC siRNA, or co-transfected with miR-29b mimics and pc-DNA3.1-LASP1 plasmid, or miR-29b mimics and blank pc-DNA3.1 vector, respectively, using Lipofectamine 2000 (Thermo Fisher), according to the manufacture's instruction. Cells were then cultured for 48 h before the following assays.

### Bioinformatics analysis

Targetscan software (http://www.targetscan.org), Pictar (pictar.mdc-berlin.de), and MiRanda (http://www.microrna.org) were used to predicate the putative targets of miR-29b, according to the manufacture's instruction.

### Construction of recombinant vectors for luciferase reporter assay

The predicted miR-29b binding sites on the 3’-untranslated region (3’UTR) of LASP1 were cloned into the pGL3 vector (Promega Corporation, Madison, WI, USA) named pGL3-LASP1-3’UTR. The mutant miR-29b binding sites on the 3’UTR of LASP1 were constructed using a QuikChange Site-Directed Mutagenesis kit (Stratagene; Agilent Technologies, Inc., Santa Clara, CA, USA), in accordance with the manufacture's protocol, which was also inserted into the pGL3 vector and named pGL3-LASP1-mut-3’UTR.

### Cell transfection

For functional analysis of miR-29b and LASP1, AGS and BGC-823 cells were transfected with scramble miR mimic (miR-NC), miR-29b mimic, negative control (NC) inhibitor, miR-29b inhibitor, NC siRNA, LASP1 siRNA, or co-transfected with miR-29b mimic and pcDNA3.1-LASP1 ORF plasmid, using Lipofectamine 2000 (Thermo Fisher Scientific, Inc.), according to the manufacture's instruction. For *in vivo* experiment, AGS and BGC-823 cells were stably transfected with the pLVTH-miR-29b lentiviral plasmid, or with blank pLVTH vector as control group, respectively. For the luciferase reporter assay, AGS and BGC-823 cells were co-transfected with 500 ng pGL3-LASP1-3’UTR or pGL3-LASP1-mut-3’UTR plasmid, and 50 nM miR-NC or miR-29b mimic, respectively, using Lipofectamine 2000 (Thermo Fisher Scientific, Inc.), according to the manufacture's instruction. In the control group, cells were only transfected with 500 ng pGL3-LASP1-3’UTR or pGL3-LASP1-mut-3’UTR plasmid, without transfection with miR-NC or miR-92b mimic. The luciferase activity was detected after transfection for 48 h using the Dual Luciferase Reporter Assay System (Promega), according to the manufacturer's instruction.

The article "Methylation-induced downregulation and tumor suppressive role of microRNA-29b in gastric cancer through targeting LASP1" was retracted in 2023. Reasons: duplicated images; signs of a paper mill; concerns about the data.

### Western blot

Cells were lysed in cold radioimmunoprecipitation assay buffer (Thermo Fisher Scientific, Inc.). The protein concentration was determined using the Bicinchoninic Acid Protein Assay Kit (Pierce Biotechnology, Inc., Thermo Fisher Scientific, Inc.). Protein was separated with 12% SDS-PAGE, and then transferred to a polyvinylidene difluoride (PVDF) membrane (Life Technologies; Thermo Fisher Scientific, Inc.). The PVDF membrane was then blocked in 5% non-fat milk in PBS (Life Technologies; Thermo Fisher Scientific, Inc.) containing 0.1% Tween-20 (Sigma-Aldrich, Inc.) at room temperature for 3 h. Subsequently, the PVDF membrane was incubated with rabbit anti-human polyclonal LASP1 (1:100, Abcam, Cambridge, MA, USA) or rabbit anti-human GAPDH (1:100, Abcam) primary antibodies for 3 h at room temperature. After washed with PBS for 10 min, the PVDF membrane was incubated with goat anti-rabbit secondary antibody (1:10000, Abcam) at room temperature for 1 h. After washed with PBS for 10 min, the protein bands were detected using the Enhanced Chemiluminescence Western Blotting Kit (Pierce Biotechnology, Inc.; Thermo Fisher Scientific, Inc.), according to the manufacturer's protocols, and then quantified using Image Lab analysis software 3.1 (Bio-Rad Laboratories, Inc., Hercules, CA, USA). GAPDH was used as the internal reference.

### MTT assay

An MTT assay was used to examine cell proliferation. AGS and BGC-823 cells (5×10^4^ per well) were plated into a 96-well plate and cultured at 37°C with 5% CO_2_ for 12, 24, 48 or 72 h. Subsequently, 20 μl MTT (5 mg/ml, Life Technologies; Thermo Fisher Scientific) was added. Following incubation at 37°C for 4 h, 150 μl dimethyl sulfoxide (DMSO, Thermo Fisher Scientific) was added. Following incubation at room temperature for 10 min, formazan production was detected by determining the optical density at 570 nm using a Multiskan FC enzyme immunoassay analyzer (Thermo Fisher Scientific, Inc.).

### Tumor growth *in vivo*

Male BALB/C-nu/nu nude mice (10 weeks) were maintained under pathogen-free condition at the Animal Center of Central South University. The mice (n=5 in each group) were injected subcutaneously in the dorsal flank with 1×10^7^ AGS and BGC-823 cells transfected with pLVTH-miR-29b lentiviral plasmid or blank pLVTH lentiviral plasmid. On 60 days after tumor implantation, all mice were sacrificed. Tumor weight and volume were also recorded. Tumor volume was calculated by using the formula V (mm^3^) = 0.5×a×b2 (a maximum length to diameter, b maximum transverse diameter).

The article "Methylation-induced downregulation and tumor suppressive role of microRNA-29b in gastric cancer through targeting LASP1" was retracted in 2023. Reasons: duplicated images; signs of a paper mill; concerns about the data.

### Wound healing assay

AGS and BGC-823 cells were cultured to confluence, and the wound was created with a plastic scriber. Then, cells were washed and incubated in serum-free DMEM at 37°C for 24 h. After that, the medium was replaced with DMEM with 10% FBS, and then cultured at 37°C for 48 h. The wounds were observed under a microscope (Nikon, Tokyo, Japan).

### Transwell assay

Transwell assay was conducted to examine the cell invasive capacity by using the 24-well transwell chamber (Chemicon, USA) pre-coated with Matrigel (Chemicon, USA). In briefly, AGS and BGC-823 cell suspension was added in the upper chamber, and 300 ul of DMEM with 10% FBS was added into the lower chamber. After incubation at 37°C for 24 h, those non-invading cells on the interior of the inserts were removed using a cotton-tipped swab. Cells on lower surface of the membrane was stained with gentian violet (Sigma), and then rinsed by water, and dried in air. Invading cells were counted under a microscope (Olympus, Tokyo, Japan).

### Statistical analysis

Data were expressed as the group means ± standard error of the mean and analyzed using Student's *t* test for two-group comparisons and one-way analysis of variance for multiple-group comparisons. The association of gene expression or methylation with clinical characteristics in gastric cancer was analyzed using chi-square test. Survival curves were determined by the Kaplan-Meier method. Multivariate analysis was performed to assess the relative influence of prognostic factors on overall survival using the Cox proportional hazards model with a forward stepwise procedure. P value less than 0.05 was considered significantly different.

## Abbreviations

LASP1: LIM and SH3 protein 1
miR: microRNA
DNA: deoxyribonucleic acid
RNA: ribonucleic acid
UTR: untranslational region
PCR: polymerase chain reaction
MTT: 3-(4,5-dimethyl-2-thiazolyl)-2,5-diphenyl-2-H-tetrazolium bromide
NC: negative control
siRNA: small interfering RNA
ORF: open reading frame
DMEM: dulbecco's modified eagle medium
